# Comparison of Arndt-endobronchial blocker plus laryngeal mask airway with left-sided double-lumen endobronchial tube in one-lung ventilation in thoracic surgery in the morbidly obese

**DOI:** 10.1590/1414-431X20176825

**Published:** 2017-12-18

**Authors:** Z.J. Zhang, M.L. Zheng, Y. Nie, Z.Q. Niu

**Affiliations:** Department of Anesthesiology, the Cangzhou Central Hospital, Cangzhou, Hebei, China

**Keywords:** Laryngeal mask airway, Arndt-endobronchial blocker, L-DLT, One-lung ventilation, Thoracic surgery, Morbidly obese

## Abstract

This study aimed to evaluate the feasibility and performance of Arndt-endobronchial blocker (Arndt) combined with laryngeal mask airway (LMA) compared with left-sided double-lumen endobronchial tube (L-DLT) in morbidly obese patients in one-lung ventilation (OLV). In a prospective, randomized double-blind controlled clinical trial, 80 morbidly obese patients (ASA I-III, aged 20–70) undergoing general anesthesia for elective thoracic surgeries were randomly allocated into groups Arndt (n=40) and L-DLT (n=40). In group Arndt, a LMA™ Proseal was placed followed by an Arndt-endobronchial blocker. In group L-DLT, patients were intubated with a left-sided double-lumen endotracheal tube. Primary endpoints were the airway establishment, ease of insertion, oxygenation, lung collapse and surgical field exposure. Results showed similar ease of airway establishment and tube/device insertion between the two groups. Oxygen arterial pressure (PaO_2_) of patients in the Arndt group was significantly higher than L-DLT (154±46 *vs* 105±52 mmHg; P<0.05). Quality of lung collapse and surgical field exposure in the Arndt group was significantly better than L-DLT (effective rate 100 *vs* 90%; P<0.05). Duration of surgery and anesthesia were significantly shorter in the Arndt group (2.4±1.7 *vs* 3.1±1.8 and 2.8±1.9 *vs* 3.8±1.8 h, respectively; P<0.05). Incidence of hoarseness of voice and incidence and severity of throat pain at the post-anesthesia care unit and 12, 24, 48, and 72 h after surgery were significantly lower in the Arndt group (P<0.05). Findings suggested that Arndt-endobronchial blocker combined with LMA can serve as a promising alternative for morbidly obese patients in OLV in thoracic surgery.

## Introduction

Management of one-lung ventilation (OLV) continues to be a challenge in clinical practice (1). A double-lumen endobronchial tube (DLT) or a bronchial blocker is usually used to achieve one-lung ventilation (OLV) in thoracic surgeries (2). However, DLT is not easy for nasal intubation in some cases due to its large outer diameter and distal curvature (3), particularly in patients with difficult airways (Mallampati grade view 3 or 4), restricted mouth opening and limited neck extension, as it is bulkier and more rigid than a single-lumen endotracheal tube (4,5). Distortion of the tracheobronchial tree would cause difficulties in placement of a DLT. An Arndt bronchial blocker might be better in such cases.

Obese patients are known to have increased risk of complications in airway management due to altered airway anatomy. Short neck, limited neck extension and fat deposition in the pharyngeal wall are some of the causative factors (6). Obese patients are also likely to have obstructive sleep apnea (7 [Bibr B08]–9). Maintenance of airway for surgical procedures is difficult due to changing in pulmonary mechanics and circulation (10,11). Increased residual gastric volumes and gastric fluid acidity increase the need for aspirations. Intubation with a DLT might be difficult due to its larger size and shape. At present, although techniques for lung isolation in thoracic surgery are increasing (12), reports on its optimal use in morbidly obese patients are still relatively scarce. A recent study by Campos et al. (13) on comparison between the use of L-DLT and Arndt blocker in lung isolation in the morbidly obese found that both techniques are clinically equivalent in terms of intubation difficulty and time for lung collapse.

Laryngeal mask airway (LMA) is a relatively new device. It is less invasive and causes less airway resistance. However, its application is still limited in OLV (14). In the present study, we compared the outcome of the combination of Arndt-endobronchial blocker and LMA with L-DLT in the morbidly obese patients in OLV in thoracic surgery. This was done by evaluating the airway establishment, ease of insertion, oxygenation, lung collapse, incidence of voice hoarseness and incidence and severity of throat pain of the patients.

We hypothesized that endotracheal intubation of the morbidly obese patients with Arndt-endobronchial blocker combined with LMA would be more feasible and yield better performance than L-DLT in OLV in elective thoracic surgery.

## Material and Methods

### Selection of patients

The protocol for clinical investigation performed in this study was approved by the Ethics Committee of the Cangzhou Central Hospital, Cangzhou, Hebei (No. 2015-063). Written informed consent was obtained from all participants. Eighty adult morbidly obese patients with a BMI >35 kg/m^2^ (age, 20–70 years; American Society of Anesthesiologists physical status I–III) who were scheduled for elective thoracic surgery from September 2015 to December 2016 were randomly assigned into 2 groups, Arndt group (Arndt-endobronchial blocker combined with LMA) and L-DLT group, with 40 patients in each group (Figure 1).

**Figure 1.** CONSORT flow diagram. Arndt: Arndt-endobronchial blocker association; L-DLT: left-sided double-lumen endobronchial tube.

Sequence generation was achieved with a computerized random number generator. Allocation concealment was achieved by using sealed opaque envelopes. All aspects of anesthetic management, including placing the tubes/devices, were taken care of by two experience anesthetists. All patients were informed before the procedure and were blinded to group allocation.

Exclusion criteria included an age of <20 years, preoperative hoarseness, mouth opening of <2.5 cm, symptomatic or untreated gastroesophageal reflux, pregnancy, surgery within >6 h.

### Methods of anesthesia

All patients were premedicated with 0.01 mg/kg intramuscular (*im*) injection of penehyclidine hydrochloride and 0.04 mg/kg of midazolam 30 min before induction of anesthesia. After arrival in the operation room, an intravenous (*iv*) cannula was placed and patients were maintained with infusion of Ringer's solution at a rate of 5 mL·kg^-1^·h^-1^. Induction of general anesthesia was achieved with 3–5 μg/kg fentanyl, 1.5–2 mg/kg propofol, and 0.1–0.15 mg/kg vecuronium. Central venous pressure of the right internal jugular vein was measured and routine monitoring of heart rate (HR), respiratory rate (RR), electrocardiography, oxygen arterial pressure (SpO_2_)_,_ oral temperature, radial artery pressure, and urine output were performed continuously.

After the patients were in full oxygen supply and complete muscle relaxation, a LMA™ Proseal (size 4 for female and size 5 for male; LMA North America, Inc., USA) was placed followed by a 9 Fr Arndt endobronchial blocker (Cook® Critical Care, USA) for those in the Arndt group. Patients in the L-DLT group were intubated with a left-sided [37–41] Fr double-lumen endobronchial tube (L-DLT; Broncho-cath™, Mallinckrodt Laboratories, Ireland). Tube sizes were determined by measurement of the width of the tracheal diameter (in mm) from the preoperative chest radiographs (15). When the Arndt blocker was in optimal position, the wire loop was removed and the wire channel was used for suction. The cuff pressure was maintained between 55 and 60 cmH_2_O with a manometer (Mallinckrodt, Germany). All patients were given 1–2 μg·kg^-1^·min^-1^ of vecuronium with intermittent intravenous injection of fentanyl and inhalation anesthesia of 1–2% isoflurane. Epidural lines were placed in all patients.

### Maintaining of patients

Accuracy of the Arndt or L-DLT was assessed by using a flexible fiberoptic bronchoscopy (FOB; BF type 3 C40; Olympus, Japan). Placements were confirmed by two experience thoracic anesthesiologists and were again checked after lateral positioning. Patients were carefully positioned for operation. The head was fixed and after turning to the lateral decubitus position, OLV was initiated.

During two-lung ventilation (TLV), patients were maintained at tidal volume (Vt) of 8 mL/kg, inspiratory/expiratory ratio (I:E) of 1:1.5, fraction of inspired oxygen (F_I_O_2_) of 0.6 and RR of 12 breaths per min. During OLV, patients were maintained at Vt of 6 mL/kg, I:E of 1:2, F_I_O_2_ of 0.6 and respiratory rate of 15 breaths per min. In order to prevent ventilation/perfusion ratio imbalance due to prolong OLV, suction was performed intermittently. Arterial blood gases were measured. Open thoracotomy or video-assisted thoracoscopic surgery (VATS) was performed. Tube/device position and adequacy of lung collapse were evaluated each 30 min during surgery.

After surgery, all patients were carefully extubated and received supplementary oxygen at 5 L/min via a facemask for 30 min. This was continued if SpO_2_ was less than 95% whilst breathing room air. For postoperative pain therapy, sufentanil and 0.25% bupivacaine were given upon request via the epidural catheter. Paracetamol and piritramide, 0.05 mg/kg intravenous, were given when analgesia was inappropriate.

### Observation and data collection

Intubation time was recorded with a stopwatch from the time when the tubes or devices passed the vocal cords until the anesthesiologists confirmed its correct placement and optimal position with FOB aid. A maximum of three placement attempts was allowed. Each attempt was defined as withdrawing the bronchial lumen of the Arndt or L-DLT into the trachea and then attempting to reposition it.

Correction of any inadequate seal of the LMA was performed. In case of inability to intubate with a DLT, a single-lumen tube and exchange catheter (Cook® Critical Care) was used to place a DLT, and the time was added to the original attempt time. Criteria used to assess malposition are as shown in Table 1.

**Table 1.** Criteria to assess endo-tracheal tube malpositions.

• Bronchial cuff of the DLT herniated above tracheal carina (more than 50% of the cuff)
• Bronchial cuff edge of the DLT not visible in the entrance of mainstem bronchus such that it would potentially occlude a secondary bronchus
• Arndt blocker or DLT in the non-targeted bronchus
• Bronchial cuff of the Arndt blocker herniated into carina (more than 50% of the cuff), or the distal tip of the blocker above tracheal carina

DLT: double-lumen endobronchial tube

Arterial blood gases, PaO_2_, PaCO_2_, and intrinsic positive end-expiratory pressure were collected during two-lung ventilation (baseline data) and 30 min after OLV.

After the pleura was opened and the lung could be seen, the quality of lung collapse was evaluated. The time for lung isolation/collapse was measured from the institution of one-lung ventilation to the time of total lung collapse. Evaluation of surgical exposure (evaluation criteria as referred to Campos et al. (16) method) were performed by two thoracic surgeons independently who were blind to the group assignment. Collapse of the lung was assessed as follows: 1) spontaneous, 2) assisted with suction, or 3) manual. The conditions of surgery were ranked as excellent, fair, or poor: 1) excellent: complete collapse with perfect surgical exposure, 2) fair: total collapse, but the lung still had residual air, and 3) poor: no collapse was achieved or partial collapse with interference in surgical exposure. At the end of surgery, the surgeons gave the overall assessment of the lung isolation. Results were recorded and the average was calculated.

An investigator blind to the group assignment of the patients asked the patients specific questions regarding postoperative hoarseness and throat pain at the post-anesthesia care unit (PACU) and 12, 24, 48, 72, and >72 h after surgery. Throat pain score assessment was performed with a numerical rating scale (NRS) ranging from 1 to 10 recorded by direct questioning of the patients. NRS=0 and NRS >0 were considered as painless and painful throat, respectively. All patients were trained on how to answer the NRS.

### Statistical analysis

Primary endpoints were the number of times the tube/devices were successfully position at the first intubation attempt, the number of malpositions, the time required to achieve optimal position verified by FOB, oxygenation, quality of lung collapse and surgical field exposure; Secondary outcome were incidence of hoarseness of voice and incidence and severity of throat pain.

The total number of patients recruited was based on research of previous studies (17,18), to allow detection of at least 2 min difference between the two groups in the time of tube or device placement, with an α of 0.05 and power of 0.80.

Data are reported as means±SD. Comparison between the two groups was performed using Student's *t*-test. P<0.05 was considered to be statistically significant. Analysis was performed using SPSS statistical software (version 19.0, SPSS Inc., USA).

## Results

No patient dropped out of the study. In the Arndt group, sizes of the single-lumen tracheal tubes for the Arndt® blocker 9 Fr were 8.0 mm ID (n=6), 8.5 mm ID (n=22), and 9.0 mm ID (n=12). In the L-DLT group, the tube sizes used were 37 Fr (n=19), 39 Fr (n=13), and 41 Fr (n=8).

### Demographic characteristics

Patients in the Arndt group and L-DLT group were equivalent in their basic characteristics with regard to age, male/female ratio, height, weight, BMI, neck circumference (NC), pre-operative spirometry results and pre-operative hemodynamic parameters (Table 2).

**Table 2.** Demographic characteristics, preoperative pulmonary functions and preoperative arterial blood gas values of the patients in the Arndt and L-DLT groups.

Variables	Arndt group (n=40)	L-DLT group (n=40)
Age (year)	59±12	60±11
Gender (M/F)	34/6	34/6
Height (cm)	166±6	165±7
Weight (kg)	114±11	115±10
BMI (kg/m^2^)	41.4±3	42.2±3
Neck circumference (cm)	44±4	45±5
FEV1 (% predicted)	78±13	79±14
FRC (% predicted)	135±18	135±19
RV (% predicted)	142±20	141±21
TLC (% predicted)	105±15	102±16
Smoking history (n)	21	20
PaCO_2_ (mmHg, room air)	39±2	40±2
PaO_2_ (mmHg, room air)	81±7	80±8
O_2_sat (%)	95.9±0.6	96.4±0.8
PEEPi (cmH_2_O)	3.1±0.2	3.0±0.4
Pre-op BP (mmHg)	135±22	133±21
Pre-op HR (bpm)	75±6	76±5
Surgery duration (h)	2.4±1.7*	3.1±1.8
Anesthesia duration (h)	2.8±1.9*	3.8±1.8

Data are reported as means±SD. n: number of patients; BMI: body mass index; FEV1: forced expiratory volume in 1s; FRC: functional residual capacity; RV: residual volume; TLC: total lung capacity; PEEPi: intrinsic positive end-expiratory pressure; Arndt: Arndt-endobronchial blocker association; L-DLT: left-sided double-lumen endobronchial tube.

* P<0.05 Arndt group compared with L-DLT group (*t*-test).

### Duration of surgery and anesthesia

The duration of surgery and anesthesia for the Arndt group was statistically shorter than the L-DLT group (2.4±1.7 *vs* 3.1±1.8 and 2.8±1.9 *vs* 3.8±1.8 h, respectively; P<0.05; Table 2).

Surgical procedures performed in the Arndt and L-DLT group are shown in Table 3. The number of thoracotomies and VATS in the two groups were not significantly different (P=0.48), nor were the numbers of left- and right-sided surgeries (P=0.36).

**Table 3.** Type of thoracic surgery and related outcomes of the 80 patients and airway parameters.

Type of procedure	Arndt group (n-40)	L-DLT group (n=40)	P value
Lobectomy			0.36
Right-sided	16	14	
Left-sided	8	10	
Pneumonectomy			
Right-sided	1	0	
Left-sided	1	2	
Upper and middle esophageal resection	14	14	
Airway parameters			
Mallampati grade	2.1±1.1	2.2±1.2	0.78
Cormack grade	2.2±1.3	2.3±1.2	0.68
Intubation attempts (n)	1.1±0.1	1.1±0.2	0.56
First attempt (n)	37	36	
Second attempt (n)	3	3	
Third attempt (n)	0	1	
Intubation duration (min)	3.3±0.4	3.4±0.5	0.84
Positioning attempts (n)	1.1±0.1	1.1±0.1	0.81
Number of malpositions (n)	3	3	
Positioning duration (min)	4.4±0.6	3.2±0.4	0.92
Adjustments (n)	0.6±0.2	0.4±0.1	0.35

Data are reported as mean±SD or number of patients. Arndt: Arndt-endobronchial blocker association; L-DLT: left-sided double-lumen endobronchial tube. Statistical analysis was done with the *t*-test.

### Number of intubation attempts

The number of intubation attempts and other airway parameters for group Arndt and L-DLT are reported in Table 3. Parameters between the two groups were not significantly different.

In the Arndt group, the size of LMA™ Proseal used was adequate with minimal secretions and without further complications. There was no dislodgement of mask, airway obstruction or pulmonary aspiration during anesthesia.

In the L-DLT group, for cases that failed to achieve successful tube intubation in the first attempt, a second or third attempt was performed. A single-lumen tracheal tube followed by insertion of an 11 Fr Cook® airway exchange catheter was used to advance a DLT without difficulties.

### Malpositions

There were 3 malpositions reported in the Arndt group and 3 in the L-DLT group in the first 30 min. This occurred when turning the patients from supine to the lateral position. For the 3 patients of the Arndt group, the tip of the blocker was dislodged above the tracheal carina, while for the 3 patients of the L-DLT group, the endobronchial cuff was herniated above the tracheal carina. All cases were repositioned with FOB aid with no further complications. The overall frequency of malpositions between the two groups was not significantly different (Table 3).

### Gas exchange data during OLV

During OLV, PaO_2_ of the patients in the Arndt group (154±46 mmHg) was significantly higher than the L-DLT group (105±52 mmHg; P<0.05) while P(A-a)O_2_ of the patients in the Arndt group (194±42 mmHg) was significantly lower than the L-DLT group (243±45 mmHg; P<0.05; Table 4).

**Table 4.** Gas exchange data of the 80 patients during OLV.

Variables	OLV	
	Arndt group (n=40)	L-DLT group (n=40)
Ppeak (cmH_2_O)	24±3	23±4
Pplateau (cmH_2_O)	16±2	15±2
PEEPi (cmH_2_O)	2.5±0.3	2.0±0.4
PaCO_2_ (mmHg)	39±5	38±5
PaO_2_ (mmHg)	154±46*	105±52
P(A-a)O_2_ (mmHg)	194±42*	243±45

Data are reported as means±SD. n: number of patients; OLV: one lung ventilation; Ppeak: peak inspiratory airway pressure; Pplateau: end-inspiratory airway pressure; PEEPi: intrinsic positive end-expiratory pressure; P(A-a)O_2:_ alveolar-arterial oxygen tension difference; Arndt: Arndt-endobronchial blocker association; L-DLT: left-sided double-lumen endobronchial tube.

* P<0.05 (*t*-test).

### Lung collapse and surgical field exposure

The time required for lung collapse was 14.8±6.2 min for the Arndt group and 17.0±6.4 min for the L-DLT group (P=0.39). Quality of lung collapse and surgical field exposure for the Arndt group was significantly better than the L-DLT group (excellent n=40, fair n=0, poor n=0 for Arndt group; excellent n=36, fair n=0, poor n=4 for L-DLT group; effective rate 100 *vs* 90%; P<0.05).

### Incidence of hoarseness of voice, incidence of throat pain and throat pain score

The incidence of hoarseness of voice and throat pain, and the mean score for throat pain among the patients in the Arndt group at PACU and 12, 24, 48, 72 h after thoracic surgery were significantly lower than the L-DLT group (P<0.05; Table 5). No incidence of hoarseness of voice and throat pain occurred after 72 h of surgery.

**Table 5.** Incidence of hoarseness of voice, incidence of throat pain and throat pain score among the 80 patients at PACU and 12, 24, 48, 72, and >72 h after thoracic surgery.

	Hoarseness of voice		Throat pain		Throat pain score by numerical rating scale (NRS)			
	Arndt (n, %)	L-DLT (n, %)	Arndt (n, %)	L-DLT (n, %)	Arndt group		L-DLT group	
					Mean	Maximum	Mean	Maximum
PACU	3 (7.5%)*	9 (22.5%)	6 (15%)*	13 (32.5%)	2*	3	5	6
12 h	4 (10%)*	12 (30%)	8 (20%)*	17 (42.5%)	3*	4	7	8
24 h	3 (7.5%)*	10 (25%)	7 (17.5%)*	15 (37.5%)	2*	3	5	7
48 h	2 (5%)*	7 (17.5%)	5 (12.5%)*	13 (32.5%)	1*	2	3	5
72 h	1 (2.5%)*	4 (10%)	1 (2.5%)*	7 (17.5%)	0.25*	1	2	3
>72 h	0 (0%)	0 (0%)	0 (0%)	0 (0%)	0	0	0	0

Data are reported as number and percentage. PACU: Post anesthesia care unit; Arndt total number of patients = 40; L-DLT total number of patients = 40. Arndt: Arndt-endobronchial blocker association; L-DLT: left-sided double-lumen endobronchial tube.

* P<0.05 *(t*-test).

## Discussion

Obesity is a worldwide health problem and the prevalence of morbid obesity is increasing over time. Thus, more patients requiring anesthesia for thoracic surgery will be overweight or obese. Obese patients are at risk for difficulties placing a DLT. For majority of cases, a left-sided DLT is preferred over a right-sided DLT due to its greater margin of safety. Increase in the NC could serves as a leading risk factor for difficult intubation (19,20), and it is neither associated with increased BMI or absolute obesity (20).

Studies found similar difficulty of intubation for both Arndt and DLT, however, DLT placements were exposed to additional risk such as potential for aspiration, progressive desaturation during the exchange and direct damage leading to tracheal or bronchial perforation or tension pneumothorax (2,21). LMA could be a primary option in case of difficult and failed airways. However, LMA alone is not able to provide OLV in thoracic surgeries. Studies showed that combination of LMA with Arndt-endobronchial blocker could provide effective surgical exposure in OLV. The technique was also associated with reduced fluctuations in hemodynamic response (14). LMA causes less airway resistance than endotracheal intubation which may, in turn lead to decreased bronchoconstrictive reflex, fewer pulmonary infections and less atelectasis (22).

Obesity is associated with restrictive lung disease due to increased intraabdominal pressure and decreased chest wall compliance (23,24). A study showed that decreases in forced expiratory volume in 1 s and forced vital capacity are inversely proportional to the increase in BMI (25). Low functional residual capacity and expiratory reserve volume contribute, respectively, to hypoventilation and poor lung collapse in OLV (26). Decrease in lung and chest wall compliance may also result in intraoperative hypoventilation during mechanical ventilation and increased work for breathing in the postoperative period when patients resume spontaneous ventilation (26).

In the present study, we compared the ease and success of placement of tube/devices in the morbidly obese patients in OLV for thoracic surgery between the Arndt and L-DLT group. In the Arndt group, selection of an appropriate LMA size is important. First, the mask should be able to provide an airtight seal during positive pressure ventilation. Second, the mask should not produce excessive pressure to the pharynx. Lastly, the mask should not be too large (27). In a study done by Voyagis et al. (28) attempting to decide whether the patient's age or weight was a better indicator for selecting the appropriate size of a laryngeal mask, it was found that the mean peak inspiratory pressure at which air leak occurred was greater using the sex-related method compared to the weight-related method. In a study by Asai et al. (27), it was found that a larger size (size 4 in females and size 5 in males) provided an airtight seal more frequently than smaller sizes, without producing a higher pressure on the pharynx. The incidence of air leak was significantly lower when a larger mask was used. Kagawa and Obara (29) proposed a formula for LMA size based on patient weight relationship.

In our study, the size of LMA used (size 4 in females and size 5 in males) was adequate to provide a proper seal for the patients. With the combination of Arndt blocker and LMA, tracheal suctioning can be performed via the internal channel of the FOB via direct visualization (14). There was seldom requirement for suctioning in patients of the Arndt group. It has been reported in a previous study that the oropharyngeal leak pressure of the LMA ProSeal was 32 cmH_2_O (range, 12–40 cmH_2_O) (14,30). In the present study, the peak airway pressure during OLV was 24±3 cmH_2_O in the Arndt group, which is far below the leak pressure of the LMA ProSeal and this is comparable with the previous study (14).

In the Arndt group, a second attempt was necessary to achieve successful intubation in 3 patients. Securing the airway with a single-lumen tracheal tube is the most important step in patients with difficult airways. This may have an advantage as it avoids the use of a tube exchanger (13).

In the L-DLT group, two or three attempts were necessary to achieve successful intubation in 4 patients. Intubation with a single-lumen tracheal tube followed by an airway exchange catheter is much easier than a standard laryngoscope with a DLT due to the larger size and shape of a DLT (31). Besides, Dhonneur et al. (32) described using a CTrach LMA as an alternative approach for morbidly obese patient.

A study by Gonzalez et al. (33) found NC >43 cm as an indicator for increased risk of difficult intubation while Neligan et al. (34) found no predictive association between NC and difficult intubation. Another study by Riad et al. (35) found BMI >50 and NC >42 cm as the independent predictors for difficult intubation and BMI >50 and male gender as independent predictors for difficult mask ventilation. In our study, the mean NC of the patients in the Arndt group and L-DLT group was 44±4 and 45±5 cm, respectively, while the mean BMI was 41.4±3 and 42.2±3 kg, respectively. In the Arndt group, the NC of the patients who failed the first intubation attempt was 45.5, 45.8, and 46.2 cm, while the BMI was 43.2, 43.7, and 44.1 kg, respectively, which was not significantly different from the other patients in the same group. In the L-DLT group, the NC of the patients who failed first intubation attempt was 45.8, 46.3, and 47.0 cm, while the BMI was 43.6, 43.9, and 44.3 kg, respectively, which was also not significantly different from the other patients in the L-DLT group.

Overall, in our study, difficult intubation was not significantly different between the groups. The findings were comparable with the previous study done for comparison between Arndt and DLT in obese (13) and normal weight (14) patients, and either with (14) or without (13) combination with LMA.

The number of malpositions was similar in both Arndt and L-DLT groups. Malpositioning might occur due to obese patients having shorter necks and decreased neck mobility than normal. With these patients, it might be difficult to support the head in the lateral decubitus position with a flex-position bed. Patients in the Arndt group required laryngeal mask manipulation resulting in the increase in the positioning duration by 1.2 min. However, the increase was not significantly different from the L-DLT group.

PaO_2_ of patients in the Arndt group was significantly higher than the L-DLT during OLV. The time for lung collapse was similar in both groups, and was comparable with the previous study done by Campos et al. (13) and Li et al. (14). Quality of lung collapse and surgical field exposure in the Arndt group was significantly better than the L-DLT group, which probably contributed to the shorter duration of surgery and anesthesia for the Arndt group.

Bronchial blockers have been considered the best device for patients with difficult airways. There is no need to replace a tube if mechanical ventilation is required (36). Risk of airway complications may increase when using a DLT compared to a bronchial blocker for achieving OLV (37). Sore throat and hoarseness of voice are among the well-known postoperative complications after tracheal intubation (38).

In the present study, the incidence of hoarseness of voice and the incidence and severity of throat pain in the Arndt group in the PACU and 12, 24, 48, and 72 h after thoracic surgery were significantly lower than the L-DLT group (P<0.05), which were consistent with previous studies (14,37). Curved endobronchial lumen and size of the L-DLT tubes could be the main risk factors for postoperative hoarseness during intubation and extubation. There was no incidence of hoarseness of voice and throat pain after 72 h of surgery.

LMA may cause laryngopharyngeal mucosal injury in a time-dependent manner. Studies found that prolonged use of LMA in pigs for <9 h was associated with no or mild changes in the laryngopharyngeal mucosa while clear signs of mucosal injury were observed after ≥12 h use (39). A previous study reported that injury scores of the bronchus and vocal cords in the DLT group were significantly higher than Arndt combined with ProSeal™, while the larynx injury score was significantly lower in the DLT group (14). In the present study, surgeries of >6 h duration were excluded to minimize risk.

The use of an Arndt endobronchial blocker may overcome some of the limitations of DLT, such as difficult airway. When applied in combination with Proseal™ LMA, the limitations of the traditional use of endobronchial blockers can be further overcome. This novel combination can be very useful in many clinical scenarios, and make thoracic anesthesia much easier (40). Combination of Arndt with LMA may exhibit more advantages over DLTs particularly in less invasive day-case thoracic surgeries, the number of which is rapidly increasing throughout the world (14). Development of newer designs of LMA would help to improve its usage and provide optimal and better benefits in the future.

In conclusion, combination of the Arndt-endobronchial blocker with LMA can be a promising alternative for morbidly obese patients in OLV for thoracic surgery with similar ease of airway establishment as L-DLT, better airway pressure, quality lung collapse and surgical field exposure, shorter duration of surgery and anesthesia, lower incidence of hoarseness of voice and less incidence and severity of throat pain.
